The article "Interpatient ECG Arrhythmia Detection by Residual Attention CNN" was published in 2022. Journal: Comput Math Methods Med.

# Interpatient ECG Arrhythmia Detection by Residual Attention CNN

**DOI:** 10.1155/2022/2323625

**Published:** 2022-04-08

**Authors:** Pengyao Xu, Hui Liu, Xiaoyun Xie, Shuwang Zhou, Minglei Shu, Yinglong Wang

**Affiliations:** ^1^Shandong Artificial Intelligence Institute, Qilu University of Technology (Shandong Academy of Sciences), Jinan 250353, China; ^2^College of Computer Science and Engineering, Shandong University of Science and Technology, Qingdao 266590, China

## Abstract

The precise identification of arrhythmia is critical in electrocardiogram (ECG) research. Many automatic classification methods have been suggested so far. However, efficient and accurate classification is still a challenge due to the limited feature extraction and model generalization ability. We integrate attention mechanism and residual skip connection into the U-Net (RA-UNET); besides, a skip connection between the RA-UNET and a residual block is executed as a residual attention convolutional neural network (RA-CNN) for accurate classification. The model was evaluated using the MIT-BIH arrhythmia database and achieved an accuracy of 98.5% and *F*_1_ scores for the classes *S* and *V* of 82.8% and 91.7%, respectively, which is far superior to other approaches.

## 1. Introduction

The latest survey statistics on global causes of mortality and disability of the World Health Organization demonstrate that cardiovascular disease (CVD) is one of the most serious diseases that threaten human health. The ECG signal reflects the electrical activity of the heart and is the primary basis for the diagnosis of CVD. With the development of computer technology, automatic arrhythmia detection technology has become a research hotspot.

Traditional machine learning approaches such as independent component analysis [1–3], principal component analysis (PCA) [4], support vector machine (SVM) [5], and K-nearest neighbor (KNN) [6] have been utilized to identify arrhythmias. However, these methods require artificial feature extraction and intervention. With the development of technology, deep learning has gradually become the mainstream method for automatic ECG classification [7]. There are mainly two kinds of deep learning approaches from the perspective of the dimension of ECG representation, i.e., one-dimensional (1-D) and two-dimensional (2-D).

Some studies exploit the original ECG signal as the model input. Although the proposed 1-D deep convolutional neural network (CNN) has achieved good classification results [8, 9], however, beat-by-beat classification cannot be achieved due to the fixed time window size. Lin et al. [10] proposed a method based on normalized and nonnormalized RR intervals that extract ECG morphology by wavelet analysis and linear prediction model, but this method requires lots of signal preprocessing and has low prediction accuracy. Llamedo and Martínez [11] proposed a method based on a linear classifier and a clustering algorithm; however, the clustering algorithm cannot effectively represent class at the edge, making more likely arrhythmia misjudgment. In addition, the abovementioned 1-D studies also introduced a small degree of preprocessing.

The article "Interpatient ECG Arrhythmia Detection by Residual Attention CNN" was published in 2022. Journal: Comput Math Methods Med.

The ECG signal can also be converted from one dimension into two dimensions in various manners, such as frequency spectrum and time-frequency images. Al Rahhal et al. [12] use the continuous wavelet transform (CWT) to generate time-frequency information, then migration learning. However, denoising and data augmentation operations reduce model efficiency. Xia et al. [13] use the heartbeat extraction method to convert multiple signals contained within 5 s into an image. However, the proposed structure not only limits the effect of the model due to the immutability of the short-time Fourier transform window but also easily causes misjudgment of normal data in verification because as long as one of the multiple heartbeats contained in the image is abnormal, the entire image will be marked as abnormal. Li et al. [14] exploited three distinct types of wavelet transforms paired with CNN to create a depth technique for automatically distinguishing time-frequency images, which identified ventricular ectopic heartbeat (*V*) as more than 97%; however, preprocessing operations such as noise reduction increase the complexity of the model. Salem et al. [15] utilized DenseNet to classify ECG spectra from the perspective of transfer learning, but it also has the same risk of misjudgment as [13]. But in terms of overall performance, the 2-D ECG data is weaker than the 1-D signal noise interference, which has also been proved in the research [16, 17].

In order to solve the problems of cumbersome preprocessing and difficult beat-by-beat classification in the above research, inspired by structural variants such as fully convolutional network, U-Net, residual network, and attention mechanism [18–27] that have been successfully used in various tasks (such as natural image classification and medical image segmentation), this paper proposes an RA-CNN model for the classification of arrhythmia between patients. Firstly, the CWT is used to convert the ECG heartbeat into an image and classes with much fewer samples are enhanced by data augmentation techniques. Secondly, the attention mechanism and residual skip connection are integrated into the U-Net which is called residual attention U-Net (RA-UNET). Finally, the RA-CNN constitutes by a skip connection between the RA-UNET and a residual block. We trained and tested the models on the MIT-BIH database, and the final experimental results demonstrate the superiority of the proposed method.

The article "Interpatient ECG Arrhythmia Detection by Residual Attention CNN" was published in 2022. Journal: Comput Math Methods Med.

The main advantages of the proposed method are summarized as follows:

1. The converted 2-D ECG will improve the effective area that the model can learn and use data enhancement methods to make up for the deficiency of waveforms [28]. The data enhancement on 1-D ECG may change its time domain information, but this problem does not exist in 2-D images
2. A new residual block (R-block) with judgment branches is proposed as the basic module of RA-CNN; it judges whether to retain the original feature map and thus solves the performance degradation
3. RA-UNET integrates the “split-transform-fusion” principle, splits the feature map into two groups after each sampling operation, uses the two branches of spatial and channel generate attention weights in parallel, and then fuses the weight feature maps of the two branches together to guide model learning

The rest of this paper is organized as follows. The proposed model is discussed in detail in Section 2, followed by the experimental design and verification in Section 3. Conclusions are finally drawn in Section 4.

## 2. Methodology

### 2.1. Database

The suggested approach is trained and evaluated using the MIT-BIH arrhythmia database [29]. It was developed in collaboration between the Massachusetts Institute of Technology and Beth Israel Hospital in Boston and is now considered one of the three primary databases in academic circles. The database contains 48 Holter records from 25 men and 22 women between the ages of 32 and 89 (of which 201 and 202 are from the same male), all of which have significant variances. Each recording is a dual-channel signal with a sampling rate of 360 Hz and a length of slightly more than 30 minutes, with the *R* peak value of each heartbeat indicated.

### 2.2. Preprocessing

#### 2.2.1. ECG Heartbeat Segmentation

Because each heartbeat in an ECG has a distinct duration, the length of it segmented from an ECG is not equal. Different methods of heartbeat segmentation were employed in the literature [30–32] in the study of 2-D.

We directly used the *R* peak position in the MIT-BIH database without additional positioning and confirmed the beat length after positioning the QRS complex according to the *R* peak position [33]. *R*_current_, *R*_previous_, and *R*_last_ represent the *R* wave peaks of the currently located heartbeat and the adjacent heartbeats before and after; the *R*-*R* interval between two adjacent *R* waves is regarded as a segment. In order to fully ensure the integrity of the segmented heartbeat medical information, the middle 3/4 position of the two *R* peaks of *R*_previous_ and *R*_last_ is taken as the intercepted heartbeat length; therefore, the intercepted *n*-th heartbeat can be expressed as Formula (1) (Figure 1):

(1) $$\begin{array}{c} E_{\text{Beat}}=\frac{3\left(R_{\text{last}}-R_{\text{previous}}\right)}{4}, \end{array}$$

where *E*_Beat_ represent the extracted heartbeat, *R*_previous_ and *R*_last_, respectively, represent the abscissa values of the previous and next heartbeat of the extracted heartbeat on the coordinate axis. If the extracted heartbeat has no heartbeat *R*_previous_ or *R*_last_, the coordinates correspond to the heartbeat; then the current heartbeat will not be segmented.

The article "Interpatient ECG Arrhythmia Detection by Residual Attention CNN" was published in 2022. Journal: Comput Math Methods Med.

#### 2.2.2. Transforming the 1-D ECG into 2-D ECG

After determining the sampling length of each beat, the 1-D ECG is converted to the time-frequency domain by CWT [28]. The choice of CWT is motivated by its success at analyzing ECG signals. The dimension of this output is higher than the dimension of the input. Unlike feature reduction, overcomplete representations allow finding more robust and sparse feature representations from the data [12]. For ECG time series, its CWT relative to a given mother wavelet *E*_Beat_ is defined as follows:

(2) $$\begin{array}{c} C_{a,b}E_{\text{Beat}}\left(t\right)=\frac{1}{{\left|a\right|}^{1/2}}\int_{-\infty }^{\infty }{\text{E}}_{\text{Beat}}\left(t\right)\psi \left(\frac{t-b}{a}\right)dt. \end{array}$$

Among them, *a* and *b* are the scale and translation parameters, respectively. *E*_Beat_(*t*) is the given signal; *ψ* is the mother wavelet.

#### 2.2.3. Heartbeat Augmentation

Even in patients with arrhythmia, the majority of the swings in the ECG analysis are normal signals, leading to fewer damage data in the ECG database. The use of data augmentation techniques to boost damage data can effectively make up for the absence of training data. Decrease the danger of overfitting, and increase the algorithm's robustness.

According to the characteristics of the 2-D ECG waveform, this article will move the beat to the left and right, move up, and move down to obtain multiple enhanced heartbeat images. The signal characteristics in the original ECG can be significantly retained by using the augmented images [34–36]. Multiple focal heartbeat data can be created after performing the preceding technique on the original ECG. In Figure 2, step (i) depicts the process of turning the extracted heartbeat into an image and step (ii) depicts a portion of the data augmentation impacts.

The abovementioned heartbeat enhancement approach is utilized to improve the data in DS_1_ (introduced in detail in this work 3.1.3). Following processing, the data balance is achieved in order to properly train the RA-CNN model.  Table 1 shows the number and percentage of heartbeats before and after enhancement.

The article "Interpatient ECG Arrhythmia Detection by Residual Attention CNN" was published in 2022. Journal: Comput Math Methods Med.

### 2.3. Model Architecture

Figure 3 shows the overall flowchart of the proposed RA-CNN model to classify arrhythmia. The encoding as images module (left) is the preprocessing process in this work 2.2 to use CWT transform the 1-D ECG into 2-D ECG heartbeat. The RA-CNN model (middle) is designed to learn 2-D ECG features so as to transform it to the forms that easy to classify. The arrhythmia prediction module (right) realizes the classification in terms of the output of RA-CNN according to arrhythmias in the AAMI standard.

The RA-CNN model consists of three parts: top layer, middle layer, and bottom layer (as shown in Figure 4). The left part of the top layer uses conv2d, avg pooling, and R-block to perform a certain degree of feature reduction on the 2-D ECG image, which is conducive to reducing the size of the input (record the output as initial feature map) and expanding the receptive fields. The right part of the top layer reduces the image dimension to 1 × 1 in order to classify by multiple consecutive R-block and avg pooling. The skip connection in the top layer is to connect the initial feature map and the output features of the other two layers. In the middle layer, the initial feature map passes through only an R-block and then connects with the output of the bottom layer. The bottom layer is residual attention U-Net (RA-UNET) which is an hourglass structure from top-to-bottom to bottom-to-top, i.e., from downsampling to upsampling; the downsampling is achieved by R-block that extracts the essential features from high-dimensional images and upsampling to be done by bilinear interpolation. A-block is applied after each downsampling and upsampling to intensify the output by generating the attention weight distribution, so that the model can efficiently focus on the appropriate area of the ECG feature. At the same time, each output of downsampling is used as a carrier to save the characteristics of the feature map via the skip connection with the output of the upsampling in the same size, which prevents inaccurate feature reconstruction. The number of image channels and size changes in the RA-CNN model structure are shown in Table 2.

1. Residual block (R-block): it is an encapsulated residual module with several convolution layers as the network infrastructure; it performs general feature learning operations or dimensionality reduction operations (such as 2.3.1).
2. Residual Attention UNET (RA-UNET): it includes a complete downsampling and upsampling process through the hourglass structure; the module has fully learned the inherent characteristics of 2-D ECG. RA-UNET converts the intrinsic feature map output of each upsampling into an attention mask to guide the feature learning of the model through skip connection, so that the model can suppress the worthless area of the feature map while enhancing specific important information (such as 2.3.2).
3. Attention block (A-block): channel attention and spatial attention are learned in parallel by grouping feature maps along the channel axis to achieve more accurate attention to important information areas (such as 2.3.3).

The article "Interpatient ECG Arrhythmia Detection by Residual Attention CNN" was published in 2022. Journal: Comput Math Methods Med.

#### 2.3.1. R-Block

R-block is a basic residual block with judgment branches, which is made up of three BatchNorm2d-Relu-Conv2d layers and then distributed throughout the RA-CNN model to accomplish the general function of feature processing.

Figure 5 shows the structural details of the R-block, which was inspired by the ResNet to solve the “degradation” problem caused by very deep levels and designed a structure with a judgment function (the Exit? branch shown in Figure 5), which decides whether to retain more original feature information by setting different steps and channels, so the purpose of it is to ensure that the essential characteristics of the feature map will not be destroyed to the maximum extent. Therefore, we can set appropriate parameters for different needs, followed by the residual connection.

For the input *X*_*R*_ of R-block, the expected output *R*(*X*_*R*_) can be expressed as

(3) $$\begin{array}{c} R\left(X_{R}\right)=\left\{\begin{array}{c} f_{i}\left(\theta^{T}\left(\sigma_{1}\left(X_{R}\right)\right)\right)⊕X_{R}\;\left(\text{i}\right),\\ f_{i}\left(\theta^{T}\left(\sigma_{1}\left(X_{R}\right)\right)\right)⊕f_{1}\left(\theta^{T}\left(\sigma_{1}\left(X_{R}\right)\right)\right)\;\left(\text{ii}\right), \end{array}\right. \end{array}$$

where *f*_*i*_(∙) is the *i*^th^ BatchNorm2d-Relu-Conv2d operation, *θ* is a convolution operation, *σ*_1_(∙) is a ReLU function, and ⊕ denotes the element-wise sum. In the Exit? process of judgment, when the number of input and output channels is equal or the convolution step is 1, the flow is shown in process (i) of Figure 5 and the expected output *R*(*X*_*R*_) is shown in the formula 3-(i). If not, the flow is shown in process (ii) in Figure 5 and the expected output *R*(*X*_*R*_) is shown in formula 3-(ii). Then the final output feature map *R*(*X*_*R*_) ∈ *ℛ*^*C*×*H*×*W*^.

The R-block solves the problem of degradation and gradient disappearance through the residual connection with judging branches, which improves the network performance and reduces the feature dimension by changing the number of channels or stride in the branch structure.

The article "Interpatient ECG Arrhythmia Detection by Residual Attention CNN" was published in 2022. Journal: Comput Math Methods Med.

#### 2.3.2. RA-UNET

RA-UNET is an improvement of the U-Net [18–22] by incorporating residual and attention mechanisms. RA-UNET is an encoder-decoder structure (as shown in Figure 6), which extracts high-level information based on three layers of downsampling and then reconstructs the feature by three layers of upsampling. In our design, the most significant thing is the attention block (A-block) inserted after each downsampling and upsampling, which can assist the model in accurate and efficient feature reduction and reconstruction. We will introduce its implementation in detail:

- Encoder: using max pooling to realize the resample of vital information of the input image, i.e., down sampling, at the same time, the A-block is used to strengthen the effect of key areas.
- Decoder: the upsampling operation is accomplished through the bilinear interpolation layer, which can be intuitively understood as the restoration process of the feature map. After each step of the upsampling operation, the A-block is also used to encourage the model to use the learned knowledge to learn more feature map information.
- Skip connections: in order to better train the deep network, after downsampling and completing the A-block, the R-block for feature processing not only better integrates contextual semantic features and prevents the disappearance of gradients caused by the stacking of coding layers but also acts as a carrier to save the characteristics; it can better restore the details of the same size feature map during the upsampling process, so as to improve the recognition effect of the network on the diversity of waveform changes.

The specific size changes and convolution kernel size during RA-UNET processing are shown in Table 3.

#### 2.3.3. A-Block

A-block captures remote contextual information in the spatial dimension and channel dimension, respectively. The attention mechanism is an improvement in the article [24], which is used to automatically learn and calculate the contribution of input data to output data. First, the sampled feature map is divided into *n* groups along the channel axis, and each group of features is split into two branches for channel attention and spatial attention, respectively, and then concatenates the attention results of the two branches together. Finally, the *n* groups of features are merged to obtain a feature map with the same size as the input.  Figure 7 shows in detail one group of attention mechanisms after channel grouping.

Take the feature map X ∈ *ℛ*^*C*×*H*×*W*^ as an example, which is the output after the first use of max pooling in RA-UNET. First, divide its channel dimension into *n* groups of subfeatures *X*_*i*_ ∈ *ℛ*^(*c*/*n*)×*H*×*W*^ (1 ≤ *i* ≤ *n*); then split each subfeature along the channel axis into two branches *X*_*i*1_, *X*_*i*2_ ∈ *ℛ*^(*c*/2*n*)×*H*×*W*^ (1 ≤ *i* ≤ *n*); hence, the channel attention is performed on the first branch to embed global information and generate channel statistical attention weight distribution by average pooling layer and softmax function. Then, the channel attention weight distribution is imposed on *X*_*i*1_ to help model focus on the distinct channel, followed with the residual connection. The final output feature map *X*_*i*1_′ of the channel attention can be realized as follows:

(4) $$\begin{array}{c} X_{i1}^{\prime }=\left(\sigma_{2}\left(W_{1}∙AVG\left(X_{i1}\right)+b_{1}\right)⊗X_{i1}\right)⊕X_{i1}. \end{array}$$

Among them, *σ*_2_(∙) represents the softmax function, AVG (∙) is the average pooling operation, *W*_1_ ∈ *ℛ*^(*c*/2*n*)×1×1^ and *b*_1_ ∈ *ℛ*^(*c*/2*n*)×1×1^ are parameters used for scaling and translation, and ⊗ stands for matrix multiplication.

The article "Interpatient ECG Arrhythmia Detection by Residual Attention CNN" was published in 2022. Journal: Comput Math Methods Med.

Next, the spatial attention is performed on the second branch to generate the spatial attention map which pays more attention to the important pixel area that stands for the principal character of the feature map. What is different from channel attention is that *X*_*i*2_ obtained the spatial attention weight distribution via group normalization, and other operations are similar. The final output feature map *X*_*i*2_′ of spatial attention can be achieved as follows:

(5) $$\begin{array}{c} X_{i2}^{\prime }=\left(\sigma_{2}\left(W_{2}∙\text{G}N\left(X_{i2}\right)+b_{2}\right)⊗X_{i2}\right)⊕X_{i2}. \end{array}$$

Among them, *GN*(∙) denotes the group normalization, *W*_2_ ∈ *ℛ*^(*c*/2*n*)×1×1^ and *b*_2_ ∈ *ℛ*^(*c*/2*n*)×1×1^ are model parameters need to be trained.

In order to maintain the consistency of channel dimensions after the attention operation, the channel attention feature map and the spatial attention feature map are spliced along the channel axis.

(6) $$\begin{array}{c} X_{i}^{\prime }=\text{Concat }\left\{X_{i1}^{\prime },X_{i2}^{\prime }\right\}, \end{array}$$

where Concat {∙} denotes the dimension concatenating operation and *X*_*i*_′ ∈ *ℛ*^(*c*/*n*)×*H*×*W*^ (1 ≤ *i* ≤ *n*).

Finally, after *n* groups of feature maps are also aggregated along the channel dimension, the final attention feature map containing the weight coefficient is generated: *X*′ = Concat {*X*_1_′, *X*_2_′, ⋯*X*_*n*_′}.

#### 2.3.4. Arrhythmia Predication

Finally, the RA-CNN model uses a fully connected layer to perform a fully connected operation on the learned attention feature map to achieve arrhythmia classification.

The article "Interpatient ECG Arrhythmia Detection by Residual Attention CNN" was published in 2022. Journal: Comput Math Methods Med.

## 3. Experimental Design

### 3.1. Experimental Setup

#### 3.1.1. Experimental Environment

The data preparation section of this paper is done on an i7-10700K processor. The experiment was done with the NVIDIAA 100 graphics card and completed on the Ubuntu 18.04.3 operating system. Run PyTorch, and then use WFDB packet to process the ECG signal.

#### 3.1.2. Classification Standard of ECG

This study used the widely used [37–42] American progressive association AAMI to develop medical device ANSI/AAMI EC57:2012 standards to classify arrhythmias. Arrhythmias are divided into five classes, as shown in Table 4.

#### 3.1.3. Database Set

The data from MIT-BIH is used to train the model in this work. This paper strictly follows the AAMI classification standard, ignoring 4 records with severe noise among the 48 records. For the remaining records, an interpatient division scheme proposed in [37–42] is used. Divide into training set (DS_1_) and test set (DS_2_). DS_1_ contains 22 records for training and parameter determination. DS_2_ is only used as a test set for final performance evaluation. Using this partitioning method, there is no need to worry about including the same patient's heartbeat in both training and test sets. The number of heart beats after division is shown in Table 5.

#### 3.1.4. Training Parameter Setting

The learning rate is a key training parameter in the proposed RA-CNN model. We optimize the parameters in order to train the model for the best performance in arrhythmia classification.

We set the initial learning rate to 0.001 and drop to the original 0.1 every 20 epochs. In order to reduce the memory, use a smaller batch size for training, and set the batch size to a small batch of 16; the loss function uses cross entropy error, and the optimization function uses Adam.

#### 3.1.5. Evaluation Metrics

This study utilized the MIT-BIH arrhythmia database to evaluate the RA-CNN model according to the AAMI standard in order to test its performance. These indicators have also been employed extensively in research [37–42]: classification accuracy (Acc), sensitivity (Sen), positive prediction rate (Ppr), and *F*_1_-score.

Acc is the proportion of correctly classified ECG samples to the total sample and is also the most commonly used evaluation index in all classification problems.

(7) $$\begin{array}{c} \text{Acc}=\frac{\text{TP}+\text{TN}}{\text{TP}+\text{TN}+\text{FP}+\text{FN}}\times 100\%. \end{array}$$

Sen only processes positive heartbeats, which means the ratio of the detected true positive heartbeats to the actual positive heartbeats.

(8) $$\begin{array}{c} \text{Sen}=\frac{\text{TP}}{\text{TP}+\text{FN}}\times 100\%. \end{array}$$

Ppr represents the proportion of positive heartbeats that are correctly detected among all positive heartbeats.

(9) $$\begin{array}{c} \text{Ppr}=\frac{\text{TP}}{\text{TP}+\text{FP}}\times 100\%. \end{array}$$

*F*_1_-score is a comprehensive evaluation index of precision rate and recall rate, used to reflect the overall situation.

(10) $$\begin{array}{c} F_{1}=\frac{2\times \text{Sen}\times \text{Ppr}}{\text{Sen}+\text{Ppr}}\times 100\%. \end{array}$$

Among the above four evaluation indicators, false positive (FP) is the number of heartbeats that are misclassified. For example, it is actually a heartbeat of class *N* but is classified into one of the classes *V*, *F*, or *S*. False negative (FN) is the number of heartbeats classified in different categories; it is also a misclassification of samples. True positive (TP) is the number of heartbeats that are correctly classified. True negative (TN) is the number of heartbeats that do not belong to a certain category and are not classified as such.

The article "Interpatient ECG Arrhythmia Detection by Residual Attention CNN" was published in 2022. Journal: Comput Math Methods Med.

### 3.2. Experimental Verification

#### 3.2.1. Analysis of the Impact of A-Block on Classification Results

Figure 8 shows the heartbeat display of channel attention and spatial attention after A-block processing in the process of using RA-UNET. A-block explores attention by assigning higher weights to pixels that are helpful for accurate classification. Therefore, as the depth of the RA-UNET deepens, the pixel area that represents the ECG curve in the feature map will become more and more obvious. The RA-UNET model will not only focus more precisely on the specific area of the lower part of the image where the waveform changes more but also filter the background information. Thereby, it can “do no useless work” and has the effect of improving the classification accuracy. In the figure, (i) shows 8 beats randomly selected from 2-D ECG, (ii) shows the visualization results output by Channel attention in A-block for the first time, and (iii) shows the output result of spatial attention structure processing. Obviously, it can be seen that (iii) pays more attention to the lower area of the image than (ii) and realizes that the large-scale, multichannel features are concentrated in the key positions of the various waveforms at the bottom of the image.

#### 3.2.2. Data Enhancement Experiment

Figures 9 and 10, respectively, show the best results of classification of classes *N*, *S*, *V*, and *F* ECG using RA-CNN when only setting variables for data enhancement. It can be found that the number of correctly classified samples after enhancement has increased compared with that before enhancement.

The article "Interpatient ECG Arrhythmia Detection by Residual Attention CNN" was published in 2022. Journal: Comput Math Methods Med.

Table 6 shows the evaluation results before and after data enhancement using the indicators mentioned in 3.1.5. It can be seen that with the basic settings unchanged, the average accuracy of the data enhancement method proposed in this work has increased by about 0.8%. Other indicators have also improved, so the data enhancement method proposed in this work can promote the classification results.

The final experimental results show that the model has a good classification effect on class *N* and class *V*, while the class *S* classification effect is significantly lower than the other two classes. The main reason is that the number of training samples for class *S* is significantly less than the other two categories even with data enhancement. The second is that the similarity of the waveforms between class *S* and class *N* is extremely high, causing the two types of samples to overlap more in the distribution, and the classification effect is not ideal.

#### 3.2.3. Ablation Study

It has been proved by 3.2.2 that the data enhancement method proposed in this work is effective. Therefore, the effectiveness of the proposed two basic structures of R-block and A-block is verified in the same situation using the enhancement method proposed in this work.  Table 7 presents the results of our ablation experiments.

First of all, we verify the influence of the R-block module on the model effect. We use conv2d (the same as the conv2d used in R-block) to replace the R-block that implements the downsampling effect in the model and remove the R-block that implements the general feature processing function. The final implementation result (as shown without R-block) shows that the classification effect would be reduced without R-block, so R-block is effective for improving the classification effect.

Secondly, we verify the effectiveness of A-block. First, remove the A-block used to capture contextual information after the sampling step. The experimental results show that A-block also has a greater impact on the accuracy of classification. Then, the effectiveness of the channel attention branch and the spatial attention branch in the A-block were verified. By removing the two branches, respectively, it was proved that the two branches also have an important influence on the context information capture of the A-block, through the evaluation of the three classes of *N*, *S*, and *V* through the general evaluation indicators.

Finally, we verify the effectiveness of the skip connection used in the top layer and middle layer. The reason why the skip connection structure is used is that RA-UNET uses the function of ReLU in the feature learning process, which will make the output result between (0, 1); therefore, the value of the feature map will decrease over time as a result of a series of feature learning operations, resulting in unsatisfactory learning effects. Through the addition of the relatively original features of the top layer and middle layer, it is possible to minimize the loss of important information without attention learning. The final experimental findings also fully validate the efficacy of this step.

The article "Interpatient ECG Arrhythmia Detection by Residual Attention CNN" was published in 2022. Journal: Comput Math Methods Med.

#### 3.2.4. Performance Comparison

We compared this study to similar studies in recent years to verify the advanced nature of RA-CNN in the classification of arrhythmia.  Table 8 displays the research findings based on data from the MIT-BIH arrhythmia database, which has been segmented in the same way as this paper. Each method's name, the year it was proposed, and its performance in the classification task are listed in the table.

[38] used traditional methods for classification research, introduced 60 features for the classification step. Not only was the preprocessing process complicated, but also the class S Ppr value was 48.8%, which is not ideal. [39] It is necessary to read multiple heartbeat features for heartbeat classification, which undoubtedly increases the amount of calculation. [40] In addition to inputting the original signal as input, the model also introduces RR interval information, which requires additional feature extraction operations, and the obtained classification effect is also worse than this study [41]. After completing the initial classification using a deep dual-channel CNN (DDCNN), it is necessary to further use the central-towards LSTM supportive model (CLSM) to distinguish classes *N* and *S*; however, the classification effect of category *S* is still unsatisfactory. [42] not only performed tedious noise reduction processing but also introduced the RR interval relationship as a feature for learning, which undoubtedly increased the difficulty of feature extraction. Compared with the above experiments, this model not only has a simple feature extraction process but also has a higher *F*_1_ value for beat-by-beat classification, which is superior in class *S* pathology identification [38–42].

## 4. Conclusion

In this work, we propose a novel and effective RA-CNN model. Experiments on arrhythmia data interpatients show that the model has a high ECG recognition ability, strong generalization, and robustness. When doctors diagnose electrocardiograms, they are mostly obtained in the form of images, and two-dimensional research is more conducive to visualization, thereby improving the efficiency of diagnosis and prevention of CVD. The data does not require any form of noise reduction operation and manual feature extraction, which avoids the loss of detailed information in the original ECG data and affects the feature extraction effect [16, 17]. The preprocessing does not need to strictly extract a single heartbeat. Even if the heartbeat is mixed with the information of the front and back heartbeats, the ECG characterization information can be better expressed through the CWT, and finally, a good classification performance can be achieved.

The article "Interpatient ECG Arrhythmia Detection by Residual Attention CNN" was published in 2022. Journal: Comput Math Methods Med.

In a further work, we will investigate the improved ECG network and further improve the classification performance of different types of diseases [43–46]. On the clinical side, we will develop an ECG system that can be deployed on wearable medical devices and automatic diagnosis algorithm, test, and improve its performance [9, 47].

## Figures and Tables

**Figure 1:** Heartbeat segmentation schematic diagram.

**Figure 2:** 2-D data generation and enhancement.

**Figure 3:** RA-CNN model training flowchart.

**Figure 4:** RA-CNN model.

**Figure 5:** R-block.

**Figure 6:** RA-UNET structure diagram.

**Figure 7:** A-block.

**Figure 8:** 2-D ECG data processing results of the two branches of A-block.

**Figure 9:** Confusion matrix without data augmentation.

**Figure 10:** Confusion matrix enhanced with data augmentation.

**Table 1:** Data comparison before and after dataset enhancement.

Database	Enhancement	Type	Number of heart beats				Total
			*N*	*S*	*V*	*F*	
MIT-BIH	Before	Amount	90042	2779	7007	802	100630
		Percentage (%)	89.48	2.76	6.96	0.80	—
	After	Amount	90042	20696	41099	8668	160505
		Percentage (%)	56.10	12.89	25.61	5.40	—

**Table 2:** The number of channels and output dimensions of each layer.

Layer name	Operate	Kernel size	Stride	Output size	Channels
Input				224 × 224	3
Top layer	conv2d	7 × 7	2	112 × 112	16
	Max Pool2d	3 × 3	2	56 × 56	16
	R-block1	$\left(\frac{\text{conv}2\text{d},1\times 1,4}{\begin{array}{c} \text{conv}2\text{d},3\times 3,4\\ \text{conv}2\text{d},1\times 1,16 \end{array}}\right)\times 1$	1 1 1	56 × 56	16
Middle layer	R-block5	$\left(\frac{\text{conv}2\text{d},1\times 1,4}{\begin{array}{c} \text{conv}2\text{d},3\times 3,4\\ \text{conv}2\text{d},1\times 1,16 \end{array}}\right)\times 1$	1 1 1	56 × 56	16
Bottom layer	RA-UNET			56 × 56	16
Top layer	R-block2	$\left(\frac{\text{conv}2\text{d},1\times 1,8}{\begin{array}{c} \text{conv}2\text{d},3\times 3,8\\ \text{conv}2\text{d},1\times 1,32 \end{array}}\right)\times 1$	1 2 1	28 × 28	32
	R-block3	$\left(\frac{\text{conv}2\text{d},1\times 1,16}{\begin{array}{c} \text{conv}2\text{d},3\times 3,16\\ \text{conv}2\text{d},1\times 1,64 \end{array}}\right)\times 1$	1 2 1	14 × 14	64
	R-block4	$\left(\frac{\text{conv}2\text{d},1\times 1,16}{\begin{array}{c} \text{conv}2\text{d},3\times 3,16\\ \text{conv}2\text{d},1\times 1,64 \end{array}}\right)\times 1$	1 2 1	7 × 7	64
	Avg Pool2d	7 × 7	1	1 × 1	64
Output				4	

The article "Interpatient ECG Arrhythmia Detection by Residual Attention CNN" was published in 2022. Journal: Comput Math Methods Med.

**Table 3:** Each layer structure and input size of RA-UNET.

Name	Layer	Kernel size	Output size	Channels
Encoder	Max Pool2d	3 × 3, stride 2	28 × 28	16
	A-block	—	28 × 28	16
	R-block	$\left(\frac{\text{conv}2\text{d},1\times 1,4}{\begin{array}{c} \text{conv}2\text{d},3\times 3,4\\ \text{conv}2\text{d},1\times 1,16 \end{array}}\right)\times 1$	28 × 28	16
	Max Pool2d	3 × 3, stride 2	14 × 14	16
	A-block	—	14 × 14	16
	R-block	$\left(\frac{\text{conv}2\text{d},1\times 1,4}{\begin{array}{c} \text{conv}2\text{d},3\times 3,4\\ \text{conv}2\text{d},1\times 1,16 \end{array}}\right)\times 1$	14 × 14	16
	Max Pool2d	3 × 3, stride 2	7 × 7	16
	A-block	—	7 × 7	16

Decoder	Upsample	Size (14, 14)	14 × 14	16
	A-block	—	14 × 14	16
	Upsample	Size (28, 28)	28 × 28	16
	A-block	—	28 × 28	16
	Upsample	Size (56, 56)	56 × 56	16
	A-block	—	56 × 56	16
	R-block	$\left(\frac{\text{conv}2\text{d},1\times 1,4}{\begin{array}{c} \text{conv}2\text{d},3\times 3,4\\ \text{conv}2\text{d},1\times 1,16 \end{array}}\right)\times 1$	56 × 56	16

Output			56 × 56	16

**Table 4:** Classification of ECG in the MIT-BIH database using AAMI standard.

Types	Contains heartbeat type
Normal (*N*)	Normal (NOR), left bundle branch block (LBBB), right bundle branch block (RBBB), atrial escape (AE), node (junction) escape heartbeat (NE)
Ventricular ectopic heartbeat (*V*)	Premature ventricular contraction (PVC), ventricular escape heartbeat (VE)
Fusion heartbeat (*F*)	Fusion of ventricular and normal (FVN)
Supraventricular ectopic heartbeat or premature heartbeat (*S*)	Atrial premature (AP), aberrant atrial premature (AaP), nodal (junctional) premature (NP), supraventricular premature (SP)
Unknown heartbeat (*Q*)	Paced (/), fusion of paced and normal (FPN), unclassified (U), undetermined (?)

**Table 5:** Interpatient dataset partitioning scheme.

Database	Datasets	Partition	Number of heart beats				Total
			*N*	*S*	*V*	*F*	
MIT-BIH	DS_1_	Training	45824	18860	37880	8280	110844
		Percentage (%)	41.34	17.01	34.17	7.47	100
	DS_2_	Testing	44218	1836	3219	388	49661
Total			90042	20696	41099	8668	160505

**Table 6:** Comparison of effects before and after data enhancement.

Enhancement	ACC	*N* (%)			*S* (%)			*V* (%)		
		SEN	Ppr	*F*_1_	SEN	Ppr	*F*_1_	SEN	Ppr	*F*_1_
Without	97.6	98.16	98.29	98.23	75.93	71.56	73.68	89.93	82.95	86.30
Proposed	98.5	98.87	98.64	98.75	83.06	82.48	82.77	93.46	90.04	91.72

**Table 7:** Data analysis of ablation experiments.

Works	ACC	*N* (%)			*S* (%)			*V* (%)		
		SEN	Ppr	*F*_1_	SEN	Ppr	*F*_1_	SEN	Ppr	*F*_1_
Without R-block	97.4	97.49	98.41	97.94	77.72	71.85	74.67	91.92	78.26	84.54
Without A-block	97.2	97.72	98.15	97.94	71.35	66.23	68.69	88.38	78.77	83.30
Without channel attention	97.7	98.18	98.21	98.20	76.68	68.84	72.61	89.84	86.35	88.06
Without spatial attention	97.5	97.95	98.08	98.02	75.44	68.40	71.74	88.75	83.51	86.05
Without top layer	96.5	96.36	97.88	97.11	74.83	64.87	69.50	90.59	72.86	80.76
Without middle layer	97.3	97.28	98.48	97.88	80.39	72.60	76.30	92.17	77.19	84.02
Proposed	98.5	98.87	98.64	98.75	83.06	82.48	82.77	93.46	90.04	91.72

The article "Interpatient ECG Arrhythmia Detection by Residual Attention CNN" was published in 2022. Journal: Comput Math Methods Med.

**Table 8:** Comparison of related experiments.

Works	ACC	*N* (%)			*S* (%)			*V* (%)		
		SEN	Ppr	*F*_1_	SEN	Ppr	*F*_1_	SEN	Ppr	*F*_1_
Dictionary (2018) [38]	95.1	90.9	99.4	94.2	80.8	48.8	60.8	82.2	85.4	83.8
DCNN (2018) [39]	94.0	90.6	98.8	94.5	82.3	38.1	52.1	92.0	72.1	80.9
MPCNN (2019)[40]	96.4	98.8	97.4	98.1	76.5	76.6	76.6	85.7	94.1	89.7
DDCNN + CLSM (2020) [41]	95.1	97.5	97.6	97.6	83.8	59.4	69.5	80.4	90.2	85.0
Linear discriminant (2021) [42]	87.3	78.7	99.3	87.8	89.4	37.5	52.9	86.5	93.0	89.6
Proposed	98.5	98.9	98.6	98.8	83.1	82.5	82.8	93.5	90.1	91.7

## Data Availability

The ECG signal data used to support the findings of this study have been deposited in the MIT-BIH Arrhythmia Database repository (https://www.physionet.org/content/mitdb/1.0.0/).
